RETRACTED

# Image Processing and Machine Learning-Based Classification and Detection of Liver Tumor

**DOI:** 10.1155/2022/3398156

**Published:** 2022-07-26

**Authors:** V. Durga Prasad Jasti, Enagandula Prasad, Manish Sawale, Shivlal Mewada, Manoj L. Bangare, Pushpa M. Bangare, Sunil L. Bangare, F. Sammy

**Affiliations:** ^1^CSE Department, VR Siddhartha Engineering College, Andhra Pradesh, India; ^2^Department of Mathematics, Vallurupalli Nageswara Rao Vignana Jyothi Institute of Engineering & Technology, Vignana Jyothi Nagar, Pragathi Nagar, Nizampet, Hyderabad, Telangana, India; ^3^Department of Electronics and Communication, Oriental Institute of Science and Technology, Bhopal, India; ^4^Department of Computer Science, Government College, Makdone (Vikram University), Ujjain, India; ^5^Department of Information Technology, Smt. Kashibai Navale College of Engineering, Savitribai Phule Pune University, Pune, India; ^6^Department of E&TC, Sinhgad College of Engineering, Savitribai Phule Pune University, Pune, Maharashtra, India; ^7^Department of Information Technology, Sinhgad Academy of Engineering, Savitribai Phule Pune University, Pune, India; ^8^Department of Information Technology, Dambi Dollo University, Dembi Dolo, Welega, Ethiopia

## Abstract

The liver is in charge of a plethora of tasks that are critical to healthy health. One of these roles is the conversion of food into protein and bile, which are both needed for digestion. Inhaled and possibly harmful chemicals are flushed from the body. It destroys numerous nutrients acquired through the gastrointestinal system and limits the release of cholesterol by utilizing vitamins, carbohydrates, and minerals stored in the liver. The body's tissues are made up of tiny structures known as cells. Cells proliferate and divide in order to create new ones in the normal sequence of events. When an old or damaged cell has to be replaced, a new cell must be synthesized. In other circumstances, the procedure is a total and utter failure. If the tissues of dead or damaged cells that have been cleared from the body are not removed, they may give birth to nodules and tumors. The liver can produce two types of tumors: benign and malignant. Malignant tumors are more dangerous to one's health than benign tumors. This article presents a technique for the classification and identification of liver cancers that is based on image processing and machine learning. The approach may be found here. During the preprocessing stage of picture creation, the fuzzy histogram equalization method is applied in order to bring about a reduction in image noise. After that, the photographs are divided into many parts in order to zero down on the area of interest. For this particular classification task, the RBF-SVM approach, the ANN method, and the random forest method are all applied.

RETRACTED

## 1. Introduction

The skin is the biggest organ in the human body; the liver is the second largest organ. The liver of an adult typically weighs about three pounds on average. The liver is located on the right side of the body, just behind the right lung, and is concealed by the rib cage. One lobe of the brain is located on either side of the median line that runs through the centre of the head. It reminds me of a laboratory or a chemical facility. The liver is responsible for a multitude of functions that are essential to maintaining good health. One of these functions is the transformation of food into protein and bile, both of which are required for digestion. Ingested and potentially toxic substances are flushed out of the circulation. By using the vitamins, carbs, and minerals that are stored in the liver, it degrades various nutrients that are absorbed through the gastrointestinal tract and controls the release of cholesterol. The tissues of the body are constructed from smaller structures known as cells. In the regular course of events, cells will multiply and divide in order to make new ones. When an older cell or one that has been damaged needs to be replaced, a new cell must be synthesized. In other cases, the procedure ends up being a complete and utter disaster. The tissues of dead or damaged cells that have been eliminated from the body might give rise to nodules and tumors if they are not eliminated. There are two types of tumors that can develop in the liver: benign and malignant. Malignant tumors provide a greater risk to one's health than benign tumors [1]. Liver CT scan image is shown in Figure 1.

According to the World Health Organization (WHO), liver cancer is the third most common cause of death in the world today. Cancer, in general, is one of the top causes of death. It would be helpful for oncologists to be able to segment liver tumors in order to check that there have been any changes in the size of the tumor. These data might be used to evaluate how effective the treatment is working for the patient and to determine whether or not any modifications are necessary. The categorizing of medical images is one of the most essential components of a well-developed system for the retrieval of medical pictures. When working with a significant volume of medical image data, it is very necessary to make use of the appropriate classification models. Computer tomography is utilized in the clinical identification process to provide assistance to radiologists in the detection of aberrant changes. CT imaging can give information that assists in medical diagnosis by allowing different types of tissues to be identified depending on the grey levels of the picture [2, 3].

RETRACTED

Cancer is frequently the main cause of death in countries with high standards of living. The classification of cancer in clinical practice is dependent on clinical and histological data, both of which have the potential to provide erroneous or incomplete findings. The liver, which is located in the upper abdomen, is an organ that processes food and removes waste from the bloodstream. It is responsible for digesting. If there are an abnormally high number of cells that need to be eliminated in the liver, a growth or tumor may develop in that organ. Since benign tumors do not develop into cancer, medical professionals remove them. After being medically removed, benign tumors almost never return to their original location [4, 5].

When the blood vessels contained inside a haemangioma become deformed and obstructed with blood, the condition is referred to be a tumor. Cancer is a progressive disease that destroys cells throughout the body. Cells are its primary target. Hepatocytes, which are liver cells and the most common starting point for primary liver cancer, are responsible for the development of the vast majority of these tumors. The most common starting point for primary liver cancer is in the hepatocytes. Hepatocellular carcinoma, also known as malignant hematoma, is a kind of cancer that may emerge in the liver. This type of cancer is also known as hepatocarcinoma.

Ultrasonography (US), computed tomography (CT), and magnetic resonance imaging (MRI) are the medical imaging investigations that are utilized the most frequently for the early detection and diagnosis of liver cancers (MRI). Because a clinician can use the CT picture to confirm the presence of a tumor as well as evaluate its size, precise position, and the degree to which the tumor interacts with the other tissue that is adjacent, CT is the tool that is most commonly used and preferred for detecting many different types of cancers, including colon cancer. Biopsies are an example of a minimally invasive operation that may be guided by CT scans. CT scans can also be used to plan and carry out radiation treatments for cancer, as well as plan and carry out other procedures [6].

In image processing, one of the most important steps is known as “smoothing out the picture.” This phase makes it easier to extract features and classify them. The analysis of biological images consequently necessitates the use of an appropriate filtering approach. It is necessary to choose the most effective liver tumor picture denoising algorithm if one wants to get outstanding results. It is possible to employ segmentation algorithms in order to eliminate unwanted elements from images of the liver. Following the steps of preprocessing and segmentation comes the step of feature extraction, which is then followed by the step of feature selection. After they have been selected, they will immediately go through the process of being categorized as quickly as possible. Denoising, segmenting, feature selection, and prediction algorithm selection are all aspects of liver tumor pictures that require more research and development [7].

RETRACTED

Literature survey section contains review of exiting methods for cancer detection. Methodology section contains a classification and detection method for liver tumors that is based on image processing and machine learning. The fuzzy histogram equalization technique is utilized during the preprocessing of images in order to reduce noise. Following that, the photos are split in order to locate the region of interest. The RBF-SVM, ANN, and random forest method are utilized here for the classification process. Results and Discussion contains the discussion related to experimental setup and various results achieved.

## 2. Literature Survey

The interpretation of medical images has been significantly impacted by both artificial intelligence and technological advancements in medical imaging processing [8]. CAD systems, which make use of computer technology to detect and categorize abnormalities in medical photos, are a popular topic of research right now and for good reason. CAD systems make use of computer technology to identify and classify anomalies in medical pictures. It is utilized by radiologists in order to identify lesions, determine the severity of a disease, and arrive at diagnostic conclusions utilizing computerized image analysis. In order to resolve a variety of diagnostic problems, computer-aided design (CAD) systems have been developed for use with digital images obtained from a variety of imaging modalities. These imaging modalities include computed tomography (CT), magnetic resonance imaging (MRI), and ultrasound.

The quality of the image is improved by the employment of techniques such as noise reduction, boosting, and standardizing during the preprocessing stage of the picture. Therefore, preprocessing is required since the quality of the input photographs will determine the effectiveness of following operations such as the determination of the ROI and the extraction of features. Prior to continuing with image processing tasks such as edge detection, segmentation, or compression, it is essential to first do noise reduction in order to significantly improve the quality of an image for display (keeping diagnostic features).

RETRACTED

With the use of a mean filter, it is feasible to give each pixel in a picture the same value as the average of the intensities that surround it [9]. It is easy to deploy and bring the diversity in a localized region down to a lower level. Gaussian noise, also known as mean square error (MSE), is perfect for this approach since it generates pictures that are both smooth and blurry. The adaptive mean filters adjust themselves locally to the characteristics of the picture in order to selectively minimize noise. They use local image statistics like the mean, variance, and spatial correlation in order to reliably detect and keep edges and other properties. This allows them to maintain the integrity of the data. Following this, a number known as the local mean is substituted for the noisy data in order to remove any lingering artefacts. Compared to its more conventional equivalents, adaptive mean filters are superior in their ability to reduce noise while simultaneously preserving the sharp edges of the signal.

When it comes to reducing noise in the probability density function that has a long tail, order-statistic filters perform exceptionally well. The median filter is part of the order-statistic filter family [10]. It blurs the image less than the average filter while maintaining the crispness of the edges. It works really well, particularly in situations where an image has granular noise.

Edge detection is utilized in the process of adjusting the direction and magnitude of the effect of the adaptive filter known as nonlinear diffusion. It may quiet the background while simultaneously bringing out the details in the edges. To remove the speckles from the image, a partial differential equation is solved, and the results are applied. Anisotropic diffusion fares exceptionally well when confronted to additive Gaussian noise. When attempting to estimate the edges of the image by using the gradient operator, it is challenging to cope with several noisy photos at the same time. To compensate for this shortcoming, a technique known as speckle reduction anisotropic diffusion [11] is utilized. In general, the values are greater near the margins, while the values are lower in areas that are more consistent. As a consequence of this, it maintains the mean in areas that are relatively consistent while simultaneously amplifying and preserving the edges in areas that are quite distinct.

The pixel values in a region are changed as a result of the repetitive application of the nonlinear geometric filter (GF), which modifies them based on their locations in relation to one another [12]. During the process of picture processing, GF not only successfully eliminates noise but also preserves important details. An adaptive method that was developed and given the name aggressive region growing filtering locates a filtering region in an image by using a homogeneity threshold for region expanding that has been correctly identified. The nonlinear median filter is used to smooth out pixels closer to the edges, whereas the arithmetic mean filter is used to smooth out parts of the image that are homogenous.

RETRACTED

You may use something called the discrete wavelet transform if you want to clean up a picture that has a lot of noise in it (DWT). Because of the wavelet transform's superior ability to compress energy, small coefficients are more likely to reflect background noise, whereas large coefficients are more likely to reflect information that is essential to understanding the image. It would appear that the coefficients that indicate qualities have a tendency to be spatially connected to one another and persist across all of the scales. Because of these qualities, DWT is an excellent candidate for denoising [13]. Wavelet shrinkage, wavelet despeckling within a Bayesian framework, wavelet filtering, and diffusion are examples of denoising algorithms that are based on wavelets.

A curvelet transform is quite similar to the wavelet transform in that it comprises frame components that are indexed by scale and position. The wavelet transform does not have these qualities, despite the fact that the curvelet pyramid does include directional parameters and a high degree of directional specificity. The use of curvelets can help minimize the amount of noise in medical photographs. Wavelets, which may be regarded of as wave atoms due to the fact that they follow the parabolic scaling of curvelets, might be utilized to perform excellent denoising on medical images [14].

In order to extract features from medical photographs, one must first recognize and choose a group of distinguishable and pertinent traits from inside the pictures. Extraction of spectral as well as spatial features, for instance, is a possibility. Following the extraction of features, it is essential to pick or reduce to a subset of the most distinguishing traits in order to maximize the accuracy of the classification while simultaneously reducing the total complexity.

During the process of classification, the extracted, selected, or reduced feature subsets are given a suspicious or not suspicious label depending on the results. The collection of qualities that a classification system contains can determine whether the classification process is supervised or unsupervised. The classification of data can be done in one of two ways: supervised or unsupervised.

RETRACTED

For instance, [15] created a hierarchical classifier called the decision tree classifier. In this classifier, attributes are compared to the data. A decision tree is a structure similar to a tree in which the nonterminal nodes indicate different attributes and the terminal modes represent different choice outcomes. The data is partitioned into the descendants of each nonterminal node using a threshold that is associated with one or more attributes. The method is finished when each terminal node has only one class of data connected with it. The decision tree may be used as a classification tool after the thresholds have been established during the training phase. The decision tree method is noticeably less complicated and more efficient than the neural network approach. Nevertheless, the construction of classification algorithms and the determination of threshold values for each nonterminal node are of utmost significance.

There are mathematical models that can imitate the massively parallel architecture of the brain in terms of how it processes information and how it learns to adapt biologically. Artificial neural networks are the name given to these types of models (ANNs). During the learning phase, the system will adjust its configuration in response to new information that comes from either the outside or the inside and is sent over the network. An ANN could contain one, two, or even many hidden layers depending on the circumstances. Each layer is composed of neuronal cells. A wide variety of ANN classifiers are utilized for the purpose of medical picture analysis [16].

Nonlinear transfer functions in the neurons of the hidden layer of a multilayer perceptron (MLP) [17] are a special kind of feed-forward network that consists of three or more layers. MLPs allow for the linking of data that is not capable of being separated linearly to training patterns. Feed-forward networks are best suited for medical imaging applications that make use of numerical inputs and outputs and pairs of input/output vectors that provide a clear basis for supervised training.

An RBF network [18] is a three-layer supervised feed-forward network that uses a nonlinear transfer function for the hidden neurons and a linear transfer function for the output neurons. To calculate a radial function of the distance between each pattern vector and each hidden unit weight vector, a Gaussian function is applied to the net input of each neuron. This is done so that the function may be determined. RBF networks are a great option for a broad variety of circumstances due to their inherent flexibility in terms of both their size and their topology.

RETRACTED

The support vector machine [19] is a supervised learning approach that seeks to determine the hyperplane that differentiates two groups of data most effectively. This is accomplished by first transforming the input data into a feature space with a higher dimension by utilizing kernel functions and then finding an optimum hyperplane inside the feature space with a higher dimension that most effectively isolates the data from one another.

## 3. Methodology

This section presents image processing and machine learning-based classification and detection of liver tumor (Figure 2). Images are preprocessed to remove noise by fuzzy histogram equalization technique. Then, images are segmented to identify region of interest. Classification is performed by RBF-SVM, ANN, and random forest algorithm.

Images are filtered in order to increase the amount of information that may be reflected or comprehended by people. This is accomplished by removing unnecessary details. When the histogram of the input picture is equalized, the outcome is an intensity distribution that is compatible with a histogram that is constant. This tactic increases the image's overall contrast on a consistent basis, particularly when the image's underlying data is already rather high contrast. This method has the potential to evenly distribute the intensity across the histogram. This is beneficial for areas with a low contrast. Equalization of histograms results in a more uniform distribution of the intensities that occur most often [20].

Before the image is segmented to acquire the desired ROI, dynamic fuzzy histogram equalization is applied to the image in order to increase its quality. They proceed to isolate the qualities that are most important from each of these components. It is the process of determining and organizing the components of a picture that are connected to one another. There are methods of segmentation that are based on the regions and edges of the data. By analyzing the intensity patterns that are surrounded by a cluster of surrounding pixels, it is feasible to discover anatomical or functional elements.

Within the context of this investigation, region-based segmentation was utilized to categorize the ROI according to its texture or pattern. The local mean is utilized as a cluster pattern in the technique known as *k*-means clustering. This technique divides the data into *k* separate clusters. The sum of the individual values obtained from each group is what will be used for this method. It uses squared Euclidean distances in order to identify the data that is the most nearby. In this procedure, the attributes that are presented are evaluated, and a single *k* group is designated to each data point based on those evaluations [21].

RETRACTED

This algorithm, known as random forest, is superior to all others. It enables precise classification of enormous volumes of data, which was previously impossible. It is a technique to group learning, and it is utilized in the context of classification and regression (also known as a closest neighbor predictor). During the process of learning, it constructs a huge number of decision trees and makes use of each one to provide output for the many classes contained in the model. It is possible to make predictions about all of the trees in a forest by employing a combination of different predictor trees, each of which is dependent on a random vector sample that has the same distribution on each tree. There is a significant amount of both variation and bias inside a single tree. The problem of excessive variance and high bias may be reduced with the help of random forest, which makes averages and seeks for a natural equilibrium between two extremes. This method is both quicker and more effective than others when it comes to categorizing [22].

Using mathematical models, it is feasible to create a simulation of the massively parallel architecture of the brain in terms of the information processing it is capable of as well as how it learns to adapt physically. Artificial neural networks are the name given to these types of models (ANNs). During the process of learning, the configuration of the system is continually modified whenever new data from within or outside the system is obtained over the network. This process occurs constantly. This type of education is known as iterative learning. Depending on the circumstances, an ANN might have anywhere from one to multiple secret levels. The exact number of these layers is never revealed. The components of each stratum are neuronal cells. In the field of medical image analysis, there is a wide variety of ANN classifiers that are employed [18].

According to [19], the objective of the support vector machine is to locate the hyperplane that differentiates two sets of data in the most effective manner. A kernel function is utilized to first transform the input data into a feature space that possesses a higher dimension and then to locate an ideal hyperplane within the feature space that possesses a higher dimension that most effectively isolates the data from one another. This procedure is repeated until the desired results are achieved. The RBF kernel function works very well with SVMs due to its adaptability.

## 4. Results and Discussion

A standard for the segmentation of liver tumors known as LiTS17 has been created [23]. The data and segmentation are made available by a number of clinical locations spread out over the world. The test data set has seventy CT scans, whereas the training data set contains one hundred thirty CT scans.

RETRACTED

In this study, the performance of a number of different algorithms is analyzed and compared based on three criteria: accuracy, sensitivity, and specificity. The results of the classifiers may be seen in Figures 3–5. When it comes to the classification of liver tumors, the accuracy and specificity of the SVM RBF algorithm are unmatched. The sensitivity of ANNs is significantly higher than that of other approaches.

(1) $$\begin{array}{c} \text{Accuracy}=\frac{\text{TP}+\text{TN}}{\text{TP}+\text{TN}+\text{FP}+\text{FN}},\\ \text{Sensitivity}=\frac{\text{TP}}{\text{TP}+\text{FN}},\\ \text{Specificity}=\frac{\text{TN}}{\text{TN}+\text{FP}}, \end{array}$$

where TP is true positive, TN is true negative, FP is false positive, and FN is false negative.

## 5. Conclusion

The liver is responsible for a wide variety of functions that are essential to maintaining good health. One of these functions is the transformation of food into protein as well as bile, both of which are essential for the digestive process. The elimination of substances can be inhaled by humans and that may be hazardous to the body. It does this by metabolizing the vitamins, carbs, and minerals that are stored in the liver, which results in the destruction of a large number of nutrients that were absorbed via the digestive system. Additionally, this process inhibits the production of cholesterol. The term “cell” refers to the very small structures that make up the body's tissues. In the natural order of things, cells must first reproduce and then divide before they can start producing new cells. When an older cell or one that has been damaged needs to be replaced, a new cell must be synthesized to take its place. In other contexts, the process is a complete and utter bust and should not be attempted. If the tissues of the cells that have died or been damaged and have been removed from the body are not eliminated, they have the potential to give rise to nodules and tumors. There are two distinct kinds of tumors that can develop in the liver: benign and malignant. The health risks posed by malignant tumors are far higher than those posed by benign tumors. This article presents a technique for the classification and identification of liver tumors that is based on image processing and machine learning. The approach may be found here. During the preprocessing stage of picture creation, a method known as fuzzy histogram equalization is utilized in order to cut down on image noise. After that, the photographs are divided into many parts in order to zero down on the area of interest. In this particular instance, the classification procedure makes use of the RBF-SVM, the ANN, and the random forest approach. When it comes to the classification of liver tumors, the accuracy and specificity of the SVM RBF algorithm are unmatched. The sensitivity of ANNs is significantly higher than that of other approaches.

RETRACTED

## Figures and Tables

**Figure 1:** Liver CT scan images.

**Figure 2:** Methodology for classification and detection of liver tumor.

**Figure 3:** Accuracy of classifiers for classification of liver tumor images.

**Figure 4:** Sensitivity of classifiers for classification of liver tumor images.

**Figure 5:** Specificity of classifiers for classification of liver tumor images.

## Data Availability

The data shall be made available on request.
